# Application of PRP in Chloasma: A Meta-Analysis and Systematic Review

**DOI:** 10.1155/2022/7487452

**Published:** 2022-04-07

**Authors:** Tinghan Deng, Fengrui Cheng, Shanshan Guo, Hongbin Cheng, Jingping Wu

**Affiliations:** ^1^Clinical Research on Skin Diseases School of Clinical Medicine, Chengdu University of TCM, Chengdu 610072, China; ^2^Department of Medical Cosmetology, Hospital of Chengdu University of Traditional Chinese Medicine, Chengdu 610072, China; ^3^Dermatology of Department, Hospital of Chengdu University of Traditional Chinese Medicine, Chengdu 610072, China

## Abstract

**Background:**

Chloasma is a common skin pigment disorder. Treatment of chloasma has been challenging, often unsatisfactory, and difficult to avoid recurrence. PRP is a new treatment for chloasma, but there is no consensus on its use. Lingyun Zhao's team recently reported a systematic evaluation and meta-analysis of the efficacy and safety of PRP in the treatment of chloasma, which is consistent with our ideas, but we will elaborate on the application of PRP in chloasma from a deeper and more comprehensive perspective. Before we started this study, we had registered with Prospero as CRD42021233721.

**Methods:**

The authors searched the public medical network, MEDLINE, EMBASE, Cochrane Central Register of Controlled Trials, ScienceDirect, Scopus, and Science Network. The clinical trials registry ClinicalTrials.gov databases were searched for relevant publications to June 2021. The results showed the area and severity of chloasma (MASI) or revised MASI (mMASI) score.

**Results:**

Three RCTs, one nonrandomized controlled study, and four were prospective before and after self-controlled studies met the inclusive criteria. Intradermal PRP injections significantly improved chloasma as indicated by the significant decrease MASI (average balance -6.71, 95% CI -8.99 to -4.33) and mMASI scores (average balance -2.94, 95% CI -4.81 to -1.07). The adverse reactions were mild, and there were no significant long-term adverse events. *Conclusive*. The data can reflect the effectiveness and safety of PRP therapy for chloasma. RCTs are needed to determine effective treatment parameters, and long-term follow-up should be included to better clarify the efficacy and side effects of PRP in treating chloasma.

## 1. Background

Chloasma is a pigmentation disorder that mostly affects women's faces. The cheeks, forehead, chin, lips, and neck are the most common areas exposed to the sun, but other areas are not uncommon [1]. The main clinical manifestation of brown facial patches has a significant impact on the patient's appearance and quality of life [2]. It is a disfiguring dermatosis that affects a large number of people all over the world, and it is difficult to treat because the pathogenesis is still unknown [3]. Many studies have recently confirmed that contraceptive pills, ultraviolet radiation, genetic predisposition, and sex hormone levels are all strongly linked to the occurrence of chloasma. In addition, skin destruction, barrier vascular factors, and inflammatory factors all play a role in chloasma pathogenesis. Drug therapy, chemical peeling, and laser are the most commonly used treatment methods today. Despite the fact that there are numerous ways to treat chloasma, data obtained through general methods cannot reach the ideal state. Because of its recurrence, chloasma can cause complications like irritation, excessive pigmentation after inflammation, and excessive pigmentation after rebound, making it an unsolvable problem in the field of beauty [4].

The main problems to be solved in chloasma are facial pigmentation and pigmentation after drug treatment. As a new technique used in dermatology and plastic surgery, PRP has been confirmed in the latest studies in its potential role in pigmented dermatitis. PRP is an autologous blood product defined as a platelet concentrate obtained by centrifuging blood to a concentration 3 to 5 times above the basal platelet concentration [5]. As for the mechanism of PRP in the treatment of pigmentation diseases such as chloasma, the present research can be divided into three aspects [6]. On the one hand, the key elements of platelets are contained in alpha particles. Alpha-granules contain more than 30 cytokines and growth factors. These include PDGF, TGF-*β*1 and *β*2, EGF, and MGF [7]. Of these, the most important reduction in pigmentation is TGF-*β*1 [8]. It has already been shown to reduce melanogenesis by delaying activation of extracellular signal-regulated kinases [9]. On the other hand, some recent studies show that the key pathology needs to control melanin production by adjusting the activities of extracellular kinase and prostaglandin E2 (PGE2). In addition, it guides extracellular matrix remodeling, strengthens the expression of matrix metalloproteinases, eliminates extracellular matrix elements damaged by light, and stimulates fibroblast proliferation and collagen synthesis [1]. In summary, PRP can reduce pigmentation and brighten skin tone [10], which is also the primary need of patients with chloasma.

In recent years, PRP is a novel treatment option for chloasma and has shown significant clinical improvement. However, there is no consensus on its use [11]. The safety, efficacy, and prognosis of PRP have not been fully confirmed. Zhao et al. [12] recently reported a systematic review on PRP in the treatment of chloasma, which included studies without controlled experimental designs. We will elaborate on the application of PRP in chloasma under more stringent inclusion and exclusion criteria and bias evaluation and try to explore the evaluation of efficacy and safety by multiple factors including ethnic differences and pharmacological effects. This study was registered with PROSPERO as CRD42021233721.

## 2. Method

A systematic review and meta-analysis were conducted according to the PRISMA (Preferred Reporting Items for Systematic reviews and Meta-Analysis) statement [13].

### 2.1. Search Strategy

A literature search was conducted in PubMed (1966 until acquisition time), MEDLINE (1966 until acquisition time), EMBASE (1974 to until acquisition time), ScienceDirect (until acquisition time), Scopus (until acquisition time), and Web of Science (until acquisition time). From 2000 to 2021, the clinical trial registry of ClinicalTrials.gov (http://ClinicalTrials.gov/) was searched.

The analytical strategy is to fuse the terms associated with chloasma with the terms identifying platelet rich plasma. Text and mesh term searches cover the words “platelet rich plasma,” “platelet concentrate,” “melanosis,” “chloasma,” “chloasma,” “chlodue to the factma,” “plaque,” “spot,” “chlosimilar Toma,” “color,” “photo,” “stain,” “stain,” “pigment” “And word variants and similar words combined with Boolean operators” or “and.”

We will review the list of documents that have been identified for similar tests or reviews to clarify the next research ideas. A complete article attachment of references reporting potential qualified tests will be obtained. If this is not possible, we will try to contact the author of the study to get some relevant information.

### 2.2. Sample

Inclusive criteria were as follows:

1. Participants were diagnosed with chloasma.
2. Intervention was any form of platelet-rich plasma, alone or as an adjunct in chloasma.
3. Control was placebo, standard care, or alternative topical therapies.
4. Pre- and post-treatment chloasma area and severity index (MASI) or modified MASI (mMASI) scores completed by dermatologists, as well as objective skin imaging analysis data. Other valid methods of evaluating the effects of PRP therapy include physician assessment, participants' subjective self-assessments, participant-reported outcomes, or satisfaction level. Additional outcomes included adverse effects reported during and after treatment.
5. Study type was RCTs. Without a random trial, well-designed non-RCTs and prospective before-and-after self-control research will be regarded as a narrative embodiment of the present facts.

### 2.3. Study Quality and Risk of Bias Assessment

Two authors independently assessed the risk of bias of each study in the field of sequence generation using the criteria suggested in the Cochrane Handbook of Systematic Reviews of Interventions [14]: occupational concealment, blindness for healthcare professionals, participants and evaluators, incomplete outcome data, and other potential threats to outcomes and validity. For nonrandomized and before-and-after studies, risk of bias was assessed using the ROBINS-I bias tool [15]. The tool includes assessments in seven areas: bias due to obscure, bias in choice of study participants, bias in intervention classification, bias in expected interventions, missing data bias, outcome measurement bias, and reporting outcome selection bias.

### 2.4. Data Extraction

The data was collected and given to two reviewers to complete on their own. The discrepancy will be repaired through discussion or negotiation with the third reviewer. The following blinded and structured stratification strategy will be used by reviewers. First, the title and abstract should be filtered. Second, read the first article you chose. Third, choose research that satisfies the predetermined inclusive and exclusionary criteria. The author name, study duration, location, year of publication, journal, study design, sample, patient characteristics, dose and type of PRP used, concomitant interventions and outcomes, duration of follow-up, evidence level, and quality of research were all listed in a standard format.

### 2.5. Data Synthesis and Statistical Analysis

Results are combined unless diversity indicates that the combination is unreasonable. If some studies reported results as continuous measures, while others used dichotomous methods of the same structure, we would convert the previous results from continuous measures to binary. If results were reported at different times throughout the year, data from each time were aggregated and combined with data from other trials from similar times. After data collection is complete, the final analysis point is determined by consensus.

ReviewManager version 5.3 was used for meta-analyses. A meta-analysis was performed as suggested by the Cochrane Collaboration [16]. For continuous data with the same measurement unit, the weighted average difference and 95% confidence interval are used. For continuous data with different measurement units, the standardized average balance and 95% confidence interval are used. The difference is represented by 95% confidence interval. When there was no heterogeneousness (*I*^2^ = 0), a fixed-effects model was used. We also used a random effects model. When heterogeneousness was high (*I*^2^ ≥ 70%), except for the lowest quality studies, sensitivity analyses were performed to account for heterogeneousness and to confirm the stability of the results, with *p* ≤ 0.05 considered statistically significant.

## 3. Results

From the database, a total of 101 records were retrieved (Figure 1). Following the deletion of 66 duplicate records, 35 articles were screened based on title and abstract. There is no other literature available from other sources. Eight studies were considered appropriate and included in the qualitative meta-analysis, while three studies were included in the quantitative meta-analysis after dragging through studies that did not meet inclusive criteria. Three RCTs, one nonrandomized controlled study, and four prospective before-and-after self-controlled studies were among the studies included.

### 3.1. Characteristics of Included Studies

Tables 1 and 2 summarize study characteristics and patient demographics. A total of 8 articles published between 2017 and 2021 were included in this study, which included a total of 277 patients with chloasma. All of the study patients were adults, patient age-bracket from 20 to 58 years of age, and about 80 percent of them were women. Of the eight studies included, three were from Egypt, two were from Pakistan, one was from Thailand, and the remaining two were from India. All studies used the MASI or mMASI score to assess the severity of patients' chloasma conduct an initial assessment. Of the 8 studies, 3 had subjects with skin types III and VI, 1 had subjects with skin types II, III and VI, 1 had subjects with skin types IV and V, 1 had subjects with skin types III and V, and the other 2 were not mentioned. In 4 of the studies, the type of chloasma in patients was epidermal and mixed, while the remaining 4 were not mentioned. The mean follow-up time of patients was 97 days (range 14–180 days). All studies have demonstrated the significant efficacy of PRP in the treatment of chloasma. The specific quality results of RCT and non-RCT studies are shown in Figure 2 and Table 3.

## 4. MASI

Four of the eight included studies comparing the MASI between experimental (PRP treatment) group and control group were reviewed [1, 3, 18, 20]. The baseline MASI were comparable between experimental and control groups in all included studies (*p* > 0.05). In MASI, the random-effect model showed significant differences between the experimental group and the control group (average balance −6.71, 95% CI −8.99 to −4.33; *p* < 0.05; *I*^*2*^ = 55%) (Figure 3).

### 4.1. mMASI

Four studies comparing the mMASI between experimental (PRP treatment) group and control group were enrolled in the meta-analysis [3, 4, 18, 19]. The baseline mMASI were comparable between experimental and control groups in all included studies (*p* > 0.05). A REM yielded a significant difference in mMASI between experimental and control groups (average balance −2.94, 95% CI −4.81 to −1.07; *p* < 0.05) (Figure 4). The heterogeneousness was substantial (*p* < 0.05; *I*^2^ = 87 percent). The study by Sirithanabadeekul et al. [4] was conducted in Thailand, whereas other studies were conducted in Egypt [3, 18, 19]. The racial difference may account for the heterogeneousness. The heterogeneousness decreased from 87% to 26%, and the average balance increased slightly to −3.66 (95 percent CI −4.74 to −2.57; *p* < 0.05) (Figure 5).

### 4.2. Degree of Improvement

A description of the extent of improvement can be found in five of the included studies [3, 17, 19, 20] (Table 4). The degree of improvement is mainly determined by referring to the decline ratio of MASI or mMASI score; among them, the most important values as dividing stages are 0%, 25%, 50%, and 75%, respectively. In most studies, the degree of improvement was rated as follows: 0: no feedback; 1: partial feedback (decrease 0%–25%); 2: good feedback (26%–50% reduction); 3: very good feedback (51%–75% reduction); 4: near perfect (75% reduction). Among the five studies, only one study chose the decrease ratio of MASI score as the evaluation criterion. Faiz and Meng [20] found that more than 60% of patients showed fair improvement, but no patient (0%) showed excellent response. Among them, 2 studies only used the decrease ratio of mMASI score as the basis for evaluating degree of Improvement. Tuknayat et al. [17] found that more than 80% of patients had mild or greater improvement, and about 40% of patients showed significant improvement. Topical tranexamic acid alone and topical tranexamic acid combined with PRP both showed some improvement in both groups, according to Gamea et al. [19]. PRP-treated patients, on the other hand, improved significantly more than the control group. MASI and mMASI were chosen as the improvement degree evaluation indexes for the remaining two groups. Hofny et al. [3] found that both the MASI and mMASI scores decreased and that more than 80% of patients improved mildly or significantly but that the difference between two different PRP injections was insignificant. According to Adel et al. [18], clinical efficacy of PRP alone or PRP combined with IPL was improved, but there was no significant difference between the two groups.

### 4.3. Patient Satisfaction

A total of five studies reported patients' satisfaction after treatment. In two of the RCTs looking at PRP versus other therapies, patient satisfaction was significantly higher under PRP than in the control group [4, 19]. In the study of the effect of two different injection methods of PRP and the randomized controlled study examining the efficacy of PRP alone and in combination with PRP and IPL, there was no significant difference in satisfaction with the efficacy between the experimental group and the control group [3, 18]. And in another prospective before-and-after self-control studies, more than 90% of patients were satisfied with the efficacy of PRP [2] (Table 4).

### 4.4. Adverse Events

Adverse events were mentioned in 6 studies. Faiz et al. [20] found the presence of temporary transient erythema at the injection site of PRP (13% of the patients). Hofny et al. [3] noted swelling, redness, and pain at the injection site of PRP. Sirithanabadeekul et al. [4] noted bruising at the injection site of PRP (the number was not mentioned). Tuknayat et al. [2] noted xerosis and hyperpigmentation at the injection site of PRP (the number was not mentioned). Gamea et al. [19] reported hyperpigmentation (5% of the patients), erythema (50% of the patients), and pain (60% of the patients) at the injection site of PRP (Table 4). Tuknayat et al. reported xerosis (35% of the patients) and pruritus (25% of the patients) at the injection site of PRP (Table 4).

### 4.5. Other Outcomes

In the RCTs conducted by Sirithanabadeekul et al. [4] on the efficacy of PRP in the treatment of chloasma, not only were MASI and mMASI score used as the efficacy criteria, but also indicators such as melanin levels, skin wrinkle levels, and erythema levels were used. However, based on the disease characteristics of chloasma and the requirements of this study, only melanin level was included in the analysis. They found a significant drop in melanin levels in the skin of patients treated with PRP, but there was no significant change in melanin levels in the skin of patients injected with normal saline (Table 4).

## 5. Discussion

Chloasma is a common skin pigment disorder characterized by brown patches on the face, which sometimes becomes a chronic distressing condition on the patient. Chloasma is caused by a complex interplay of factors such as sunlight, endocrine, hepatopathies, ovarian tumors, parasitic infestations, cosmetics, and stressful life events in a genetically predisposed individual [21–24]. However, the exact etiology of chloasma is still not well elucidated yet.

Although there are various treatments including drug therapy, chemical peeling, laser, etc., finding a cure for chloasma has always been challenging, often unsatisfactory, and hard to avoid recurrence [24].

In order to provide a reference for clinical treatment, we conducted a systematic review and meta-analysis to assess the safety and efficacy of PRP in the treatment of chloasma. The key finding of this systematic review was that intradermal PRP injections significantly improved chloasma, as evidenced by significant decreases in MASI and mMASI scores in various patient populations over a 12-week period. The systematic analysis found no serious or significant long-term negative effects. The effectiveness and safety of PRP therapy for chloasma were also demonstrated by the reported degree of improvement and patient satisfaction in enrolled studies. The following are some of the benefits of our research: (1) we focus on the efficacy and safety of intradermal PRP injection to improve chloasma, providing clear conclusions for other clinicians; (2) The conclusions are true and reliable due to rigorous and serious inclusion and exclusion by two professionals, and reasonable and standardized inclusion of relevant research and analysis; (3) the topic and possibility of the corresponding direction are analyzed and discussed based on the relevant professional knowledge of the team.

Our discovery is in line with a few previous studies. Cayırlı et al. [5] reported a case of a 27-year-old woman who accepted three PRP injections sessions with 15-day intervals for skin rejuvenation, and regression of chloasma achieved more than 80%. Farag et al. [25] reported a case with resistant chloasma. After six sessions of PRP injection, her MASI score came down from 17.7 to 7.5, and after a three-month follow-up, no relapse of chloasma was examined. In another case report, PRP was used as an adjuvant with Q-switched Nd-YAG laser and alpha arbutin therapy with hopeful lightening [26].

PRP is a high concentration of platelet plasma. Platelets are cellular fragments of megakaryocytes of the bone marrow. They are characterized by the absence of nuclei, organelles, and three types of granules in the cytoplasm: alpha, dense, and lambda [27]. Green fluorescence can regulate the biological medium of cell turnover and regeneration, exert influence on target cells and extracellular matrix, and thus realize the stimulation of repair and tissue regeneration. At present, the most widely studied green fluorescent factors include PDGF, TGF, and vascular endothelial growth factor, insulin-like growth factor, and EGF. Among them, TGF*β* and PDGF play the biggest role in PRP treatment of chloasma. TGF-*β*1 and PDGF present in PRP could have led to chloasma reduction [15]. TGF-1 inhibits melanogenesis by downregulating the expression of the paired-box homotypic c gene of the ommatidium-associated transcription factor (MITF) promoter in a concentration-dependent manner. PDGF not only promotes collagen production, synthesis, and extracellular matrix formation, but also promotes angiogenesis, collagen, and hyaluronic acid synthesis. The rationale is that EGF reduces melanin production by inhibiting the expression of prostaglandin E2 and the activity of tyrosinase. They can further improve the pigmentation of the spots.

PRP treats chloasma not only through the action of platelets themselves, but also through biological stimulation at the time of injection. Biological stimulation can activate the anabolic function of fibroblasts and collagen production, thus restoring the metabolism and normal function of the skin [27], which also has a certain effect on delaying the process of chloasma.

PRP appears to be a potential new therapy with significant efficacy for chloasma, as a monotherapy as well as an adjuvant therapy. Gamea et al. [19] used PRP therapy in combination with topical 5% tranexamic acid, compared to topical 5% tranexamic acid monotherapy, which showed significantly better treatment results and patient satisfaction was detected in patients of combination therapy group. Adel et al. [18] compared PRP alone versus intense pulsed light (IPL) plus PRP, proving an obvious improvement of chloasma after PRP treatment (*p* < 0.05). However, no statistically significant difference was found between the two groups regarding mMASI score or patient satisfaction (*p* > 0.05).

The clinical stage and classification of chloasma can be divided into active stage and stable stage according to the results of slide pressure diagnosis, the number and morphology of inflammatory cells and dendritic cells under the reflection confocal microscope (RCM), and the changes of the number and morphology of blood vessels under the skin microscope and the erythema index. In addition, melasma was examined by slide pressure and wood lamp. Combined with its pathogenesis, melasma can be divided into four types: pigment type (m, melanin); vascular type (V, vessel); pigment dominant type (M > V); vascular dominant type (V > m). For typing treatment, simple type M: oral chloromethylnaphthoic acid, combined with fruit acid or Q-switched laser; Type V: to improve microcirculation, Nd: YAG/KTP can be used for treatment. M > V type and V > M type: both types are formed by both pigment and vascular factors. The treatment plan should take into account the inhibition of melanin production and the improvement of blood circulation. At present, PRP can not only inhibit the synthesis of melanin, but also have a variety of repair functions, such as its antibacterial or anti-inflammatory effect and skin vascular remodeling function, which play a role in a variety of main pathological and pathogenic mechanisms of chloasma. However, more and more data are needed to support and analyze whether the efficacy of PRP combined with the above treatment schemes is better.

What we can know is that chloasma is more common among Hispanic and Oriental people, but unfortunately we have not retrieved or understood the treatment of PRP in Indochina. However, there are exact reports on the efficacy of PRP for chloasma in the Middle East, India, East Asia, and other countries included in this study.

In terms of delivery methods, Hofny et al. [3] evaluated the efficacy of PRP treatment on chloasma via two different delivery methods. A statistically significant decrease was detected in both groups after treatment (*p* < 0.05), while no significant difference was found between two delivery methods.

## 6. Limitations

This review and meta-analysis established a foundation for using PRP to treat chloasma patients. It does, however, have some limitations. First, RCTs and prospective self-controlled before-and-after studies were combined, increasing the risk of choice bias. Furthermore, the current meta-analysis is constrained by a lack of high-quality studies, and biases hampered the interpretation of study findings. Furthermore, the small sample sizes and short follow-up periods in this study may have hampered the ability to detect clinically significant differences in outcome measures. Even if we use REM, the disparity in curative effect could be due to differences in research design, population, preparation technology (centrifugal/anticoagulant), treatment (volume/frequency/method), baseline patient characteristics (age, sex, skin type, or chloasma depth), and research methods.

## 7. Conclusion

To summarize, people are becoming more aware of and interested in PRP treatment for chloasma. In light of the findings discussed above, PRP therapy is a safe and effective treatment option for chloasma, regardless of the MASI or mMASI score, the degree of clinical improvement, or patient satisfaction. To establish optimal treatment parameters, more RCTs with an adequate control group, controlling for obscure factors, and larger sample sizes are required. Furthermore, the negative effects of PRP were not fully understood, limiting clinicians' use of PRP as a first-line treatment for chloasma. Long-term follow-up for effectiveness and side-effect profiles would be beneficial.

## Figures and Tables

**Figure 1:** Flow diagram of included studies.

**Figure 2:** Cochrane risk of bias assessment of RCTs [4, 18, 19].

**Figure 3:** Forest plot comparing the chloasma area and severity index (MASI) of patients accepting PRP treatment and control group. IV: interval variable, CI: confidence interval.

**Figure 4:** Forest plot comparing the modified melasma area and severity index (mMASI) of patients accepting PRP treatment and control group. IV: interval variable, CI: confidence interval.

**Figure 5:** Forest plot of sensitive analysis of the modified MASI of patients accepting PRP treatment and control group using sensitive analysis. IV: interval variable, CI: confidence interval.

**Table 1:** Characteristics of included studies.

Author, year	Study design	Location	Number assigned/evaluated	Age	Control	PRP preparation	Treatment	Treatment time	Follow-up
Hofny et al. 2019 [3]	Prospective before-and-after self-control studies	Egypt	23/23	21–50	before-and-after self-control	(1) Double centrifugation	(1) Used PRP alone	Three sessions (four-week intervals)	1 month
						(2) 10 minutes at 1600 rpm	(2) Hemi-face study		
						(3) 10 minutes at 4000 rpm	(3) Intradermal injections on the left side and microneedling before and after PRP application on the right side		
Sirithanabadeekul et al. 2020 [4]	Randomized, split-face, single-blinded prospective trial	Thailand	10/10	33–58	Intradermal normal saline injection	(1) Single centrifugation	(1) Used PRP and saline	Four times every two weeks	1 month
							(2) Hemi-face study		
						2.4 minutes at 3200 rpm	(3) Unilateral intradermal injection of PRP and the other side was injected with saline		
Tuknayat et al. 2020 [17]	Prospective before-and-after self-control studies	India	64/65	—	before-and-after self-control	(1) Single centrifugation	(1) Used PRP alone	Three sessions (four-weeks intervals)	3 months
						(2) 8 minutes at 3500 rpm	(2) Autologous PRP injections		
Mumtaz et al. 2021 [1]	Nonrandomised controlled trial	Pakistan	64/64	20–40	Intradermal tranexamic acid	(1) Double centrifugation	(1) Used PRP and tranexamic acid	Three sessions (four-week intervals)	6 months
							(2) Grouping study		
						(2) 10 minutes at 1500 rpm	(3) Experimental group: intradermal injection of PRP		
						(3) 10 minutes at 4000 rpm	Control group: intradermal tranexamic acid		
Adel et al. 2021 [18]	Randomized prospective split-face study	Egypt	20/20	—	Intradermal injection of PRP vs intradermal injection of PRP + IPL	—	(1) Used PRP and IPL	Four sessions (two-week intervals)	1 month
							(2) Hemi-face study		
							(3) One side: intradermal injection of PRP		
							The other side: intradermal injection of PRP + IPL		
Gamea et al. 2020 [19]	Randomized controlled trial	Egypt	40/40	32–58	Topical 5% tranexamic acid	(1) Double centrifugation	(1)Used PRP and tranexamic acid	Topical tranexamic acid (twice daily for 12 weeks	1 month
							(2)Grouping study		
						(2) 3 minutes at 2000 rpm	(3) Experimental: topical tranexamic acid and intradermal injection of PRP		
						(3) 5 minutes at 5000 rpm	Control group: topical tranexamic acid		
Tuknayat et al. 2021 [2]	Prospective before-and-after self-control studies	India	40/40	—	—	(1) Double centrifugation	(1) Used PRP alone	Three sessions (one-week intervals)	3 months
						(2) 10 minutes at 1600 rpm	(2) Intradermal injection of PRP		
						(3) 10 minutes at 4000 rpm			
Faiz and Meng 2018 [20]	Prospective before-and-after self-control studies	Pakistan	20/15	21–42	before-and-after self-control	(1) Double centrifugation	Intradermal injection of PRP	Five sessions (two-week intervals)	2 weeks
						(2) 3 minutes at 1500 rpm			
						(3)5 minutes at 4000 rpm			

PRP: platelet-rich plasma; IPL: intense pulse light.

**Table 2:** Demographic and clinical characteristics of participants.

Study	Gender (M/F)	Grouping	Fitzpatrick skin type	Depth	Distribution	Baseline score	Duration of illness	Triggering factor
Hofny et al. 2019 [3]	4/19	A: microneedling with Dermapen	Types III: 7	Epidermal: 18	Malar: 1	MASI:A: 6.13 ± 2.73	1–3 years: 12 patients	Sun exposure:16 Hormonal Contraception: 3
		B: microinjections using mesoneedles	Types IV: 16	Mixed: 5	Centrofacial: 22	B: 5.73 ± 2.77 mMASI:5.71 ± 2.56	˃3 years: 11 patients	Pregnancy: 4
Sirithanabadeekul et al. 2020 [4]	0/10	A: intradermal PRP	Types III: 2	Mixed: 10	—	A: 4.92 ± 0.96	—	—
		B: intradermal normal saline	types V: 8			B: 4.98 ± 0.86		
Mumtaz et al. 2021 [1]	35/29	A: intradermal PRP	—	—	—	A: 29.84 ± 5.14	A: 24.63 ± 9.87 months	—
		B: intradermal tranexamic				B: 29.56 ± 4.39	B: 23.94 ± 8.93 months	
Adel et al. 2021 [18]	0/20	A: IPL	Types II: 3	Epidermal: 6	Centrofacial: 19	MASI:16.3 ± 7.7 mMASI:	2 months-18 years	Sun exposure: 13
		B: PRP-IPL	Types III: 9	Mixed: 14	Malar: 1	A:19 ± 6.4B: 19.8 ± 5.8		Pregnancy:0
			types V: 8					
Gamea et al. 2020 [19]	0/40	A: topical 5%	Types III (A: 11 B:12)	Epidermal: (A:12 B:8)	—	mMASI:	A:12–72 months	—
		Tranexamic acid + PRP	Types IV (A: 9 B:8)	Mixed: (A:8 B:12)		A: 12.1 ± 2.9	B: 18–80 months	
		B: topical 5% tranexamic acid				B: 11.7 ± 2.98		
Faiz and Meng 2018 [20]	12/3	—	Types III: 4	—	—	MASI:	—	—
			Types IV: 11			15.71 ± 6.81		
Tuknayat et al. 2021 [2]	36/4	—	Types IV and V	Epidermal: 29	Malar: 8	mMASI:13.7	—	—
				Mixed: 11	Centrofacial: 31			
					Mandibular: 1			

^*∗*^PRP: platelet-rich plasma; IPL: intense pulse light; MASI: melasma area severity index; mMASI: modified melasma area severity index.

**Table 3:** ROBINS-I risk of bias summary for nonrandomized controlled studies and before-after studies.

Author, year	Domain						
	Obscure	Choice of participants	Classification of intervention measures	Deviations from intended interventions	Missing data	Comparison of results	Choice of the reported result
Hofny et al. 2019 [3]	Mild	Lower	Lower	Lower	Lower	Mild	Lower
Tuknayat et al. 2020 [17]	Mild	Lower	Lower	Mild	Uncertain	Mild	Uncertain
Mumtaz et al. 2021 [1]	Mild	Lower	Lower	Lower	Lower	Mild	Lower
Tuknayat et al. 2021 [2]	Mild	Lower	Lower	Lower	Lower	Mild	Mild
Faiz and Meng 2018 [20]	Mild	Lower	Lower	High	Mild	Mild	Mild

**Table 4:** Treatment outcomes of included studies.

Study	Group	MASI		mMASI		Degree of improvement *N* (%)	Patient satisfaction *N* (%)	Adverse effects *N* (%)	Other outcomes
		Before	After	Before	After				
Faiz and Meng 2018 [20]	—	15.71 ± 6.81	4.98 ± 2.13			MASI:	—	Temporary	—
						Poor (0–25% decrease) 4 (26.7)		Mild erythema: 2(13.3)	
						Fair (26–50% decrease) 9 (60)			
						Good (51–75% decrease) 2 (13.3)			
						Excellent (>75% decrease) 0 (0)			
Hofny et al. 2019 [3]	A: microneedling with Dermapen B: microinjections using mesoneedles	11.86 ± 5.25	6.96 ± 4.82	5.71 ± 2.56	2.90 ± 2.05	mMASI:	Very satisfied: 9 (39.1)	Swelling, redness and soreness	
						Excellent (>75–100% decrease): 3 (13)	Satisfied: 9 (39.1)		
						Significant (>50–75% decrease): 8 (34.8) mild (>25–50% decrease):	Slight satisfaction: 3 (13.1)		
						9 (39.2)	Unsatisfied: 2 (8.7)		
						Slight (0–25% decrease): 3 (13.0)			
						MASI:			
						Excellent (>75–100% decrease): 3 (13.1)			
						Significant (>50–75% decrease): 5 (21,7) mild (>25–50% decrease): 10 (43.5)			
						Slight (0–25% decrease): 5 (21.7)			
Sirithanabadeekul et al. 2020 [4]	A: intradermal PRP injection B: intradermal saline injection	A: 4.92 ± 0.96 B: 4.98 ± 0.86	A: 3.5 ± 0.67 B: 4.53 ± 0.96	—	—	—	From baseline to the end of treatment, the patients' satisfaction under PRP condition was significantly improved at the time of visit	Bruising	Mean melanin levels;
									A:
									Before:
									256.73 ± 17.68
									After:
									238.63 ± 16.4
									B: 246.57 ± 22.88 (before)
									249.47 ± 21.36 (after)
Tuknayat et al. 2020 [17]	—	—	—		47.3% reduction	mMASI:	—	Xerosis	
						Excellent (>75% decrease): 4 (6.25)		Hyperpigmentation	
						Significant (51–75% decrease): 21 (32.8) mild (26–50% decrease): 27 (42.1)			
						Slight (1–25% decrease): 10 (15.6)			
						No minimal (0% decrease): 2 (3.1)			
Mumtaz et al. 2021 [1]	A: intradermal platelet-rich plasma	A: 29.84 ± 5.14	A: 8.72 ± 3.40	—	—	—	—	—	—
	B: intradermal tranexamic	B: 29.56 ± 4.39	B:14.97 ± 4.33						
Adel et al. 2021 [18]	A: PPL	16.3 ± 7.7	10.9 ± 6.3	A: 19 ± 6.4	A: 14.2 ± 5.8 B: 14.6 ± 5.5	MASI:	No significant difference between both sides	—	—
	B: PRP + IPL			B: 19.8 ± 5.8		33.13% improvement mMASI:			
						No significant difference between both sides			
Gamea et al. 2020 [19]	A: topical5%	—	—	A: 12.1 ± 2.9	A: 3.6 ± 1.9	mMASI:	A:	Hyperpigmentation:	
	B: topical 5% tranexamic acid					A:	Highly satisfied: 5 (25) mildly satisfied:	A: 1 (5)	
						Excellent (75–100% decrease): 3 (15)	10 (50)	B: 2 (10)	
						Significant (50–74% decrease): 4 (20) mild (25–49% decrease): 12 (60)	Partially satisfied: 3 (15)	Erythema:	
						Slight (0–24% decrease): 1 (5)	Not satisfied: 2 (10)	A: 10 (50)	
						B:	B:	B: 0 (0)	
						Excellent (75–100% decrease): 1 (5)	Highly satisfied: 3 (5) mildly satisfied: 2 (10)	Pain:	
						Significant (50–74% decrease): 3 (15) mild (25–49% decrease): 7 (35)	Partially satisfied: 4 (20)	A:12 (60)	
						Slight (0–24% decrease): 9 (45)	Not satisfied: 11 (55)	B: 0 (0)	
Tuknayat et al. 2021 [2]	—	—	—	13.7	6.258	—	Excellent: 4 (10)	Xerosis: 14 (35)	
							Very pleased: 19 (47.5)	Pruritus: 10 (25)	
							Pleased: 16 (40)		
							Satisfied: 1 (2.5)		
							Not satisfied: 0 (0)		

PRP: platelet-rich plasma; IPL: intense pulse light; MASI: melasma area severity index; mMASI: modified melasma area severity index.

## Data Availability

All data are available upon request to the corresponding author.

## References

[1] Maryam M., Chandio T. H., Shahzad M. K., Hanif N., Anwar S., Rafique S. (2021). Comparing the efficacy of patelet-rich plasma (PRP) versus tranexamic acid (4mg/mL) as intradermal treatments of chloasma. *Journal of the College of Physicians and Surgeons--Pakistan*.

[2] Tuknayat A., Thami G. P., Bhalla M., Sandhu J. K. (2021). Autologous intralesional platelet rich plasma improves chloasma. *Dermatological therapy*.

[3] Hofny E. R. M., Motaleb A. A., Ghazally A., Ahmed A. M., Hussein M. R. A. (2019). Platelet-rich plasma is a useful therapeutic option in melasma. *Journal of Dermatological Treatment*.

[4] Sirithanabadeekul P., Dannarongchai A., Suwanchinda A. (2020). Platelet‐rich plasma treatment for melasma: a pilot study. *Journal of Cosmetic Dermatology*.

[5] Cayırlı M., Çalışkan E., Açıkgöz G., Erbil A. H., Ertürk G. (2014). Regression of Chloasma with platelet-rich plasma treatment. *Annals of Dermatology*.

[6] Tuknayat A., Bhalla M., Thami G. P. (2021). Platelet‐rich plasma is a promising therapy for melasma. *Journal of Cosmetic Dermatology*.

[7] Merchán W., Gómez L. A., Chasoy M. E., Rodríguez C. A. A., Muñoz A. L. (2019). Platelet‐rich plasma, a powerful tool in dermatology. *J Tissue Eng Regen Med*.

[8] Hofny E. R. M., Hussein M. R. A., Ghazally A., Ahmed A. M., Motaleb A. A. (2019). Increased expression of TGF-*β* protein in the lesional skins of Chloasma patients following treatment with platelet-rich plasma. *Journal of Cosmetic and Laser Therapy*.

[9] Gamea M. M., Kamal D. A., Donia A. A., Hegab D. S. (2020). Comparative study between topical tranexamic acid alone versus its combination with autologous platelet rich plasma for treatment of melasma. *Journal of Dermatological Treatment*.

[10] Lin M. Y, Lin C. S, Hu S, Chung W. H (2020). Progress in the use of platelet-rich plasma in aesthetic and medical dermatology. *The Journal of clinical and aesthetic dermatology*.

[11] Kim H., Moon S., Cho S., Lee J., Kim H. (2017). Efficacy and safety of tranexamic acid in melasma: a meta-analysis and systematic review. *Acta Dermato-Venereologica*.

[12] Zhao L., Hu M., Xiao Q. (2021 Oct). Efficacy and safety of platelet-rich plasma in melasma: a systematic review and meta-analysis. *Dermatologic Therapy*.

[13] Moher D., au fnm, Shamseer L. (2015). Preferred reporting items for systematic review and meta-analysis protocols (PRISMA-P) 2015 statement. *Systematic Reviews*.

[14] Higgins J. P., Green S. (2009). *Cochrane Handbook for Systematic Reviews of Interventions*.

[15] Sterne J. A., Hernán M. A., Reeves B. C. (2016). ROBINS-I: a tool for assessing risk of bias in non-randomised studies of interventions. *BMJ*.

[16] Higgins J., Green S. R. (2011). *Cochrane Handbook for Systematic Reviews of Interventions*.

[17] Tuknayat A., Bhalla M., Pal Thami G. (2020). Clinical efficacy of platelet rich plasma in Chloasma. *Journal of the Dermatology Nurses’ Association*.

[18] Adel S., Serri A., Abd El-Raheem T. (2021). Study of autologous platelet-rich-plasma versus its combination with intense pulsed light in treatment of Chloasma. *Dermatologic Therapy*.

[19] Gamea M. M., Kamal D. A., Donia A. A., Hegab D. S. (2020). Comparative study between topical tranexamic acid alone versus its combination with autologous platelet rich plasma for treatment of melasma. *Journal of Dermatological Treatment*.

[20] Faiz F., Meng K. (2018). Efficacy of platelet-rich plasma in the treatment of Chloasma: a pilot study. *Journal of Pakistan Association of Dermatologists*.

[21] Achar A., Rathi S. K. (2011). Chloasma: a clinico-epidemiological study of 312 cases. *Indian Journal of Dermatology*.

[22] (2014). Epidemiology of Chloasma in Brazilian patients: a multicenter study. *International Journal of Dermatology*.

[23] (2009). A global survey of the role of ultraviolet radiation and hormonal influences in the development of Chloasma. *Journal of the European Academy of Dermatology and Venereology*.

[24] Sarkar R., Ailawadi P., Garg S. (2018). Chloasma in men: a review of clinical, etiological, and management issues. *Journal of Clinical & Aesthetic Dermatology*.

[25] Farag M., Mostafa F., Gharib K. (2020). Therapeutic effect of dermapen with PRP versus dermapen with tranexamic acid. *Chloasma Cases*.

[26] Yew C. H., Ramasamy T. S., Amini F. (2015). *Response to Intradermal Autologous Platelet Rich Plasma Injection in Refractory Dermal Chloasma*.

[27] Merchán W. H, Gómez L. A, Chasoy M. E, Alfonso-Rodríguez C. A, Muñoz A. L (2019). Platelet-rich plasma, a powerful tool in dermatology. *Journal of tissue engineering and regenerative medicine*.

